This article has been retracted.

# Benefit Modeling and Analysis of Wind Power Generation under Social Energy Economy and Public Health

**DOI:** 10.1155/2022/5635853

**Published:** 2022-06-09

**Authors:** Ying Liu, Zulkefly Abdul Karim, Norlin Khalid, Fathin Faizah Said

**Affiliations:** ^1^School of Business, Jinggangshan University, Ji'an, China; ^2^Center for Sustainable and Inclusive Development Studies (SID), Faculty of Economics and Management, Universiti Kebangsaan Malaysia (UKM), Bangi 43600, Selangor, Malaysia

## Abstract

Wind is a renewable energy source. Overall, using wind to produce energy has fewer effects on the environment than many other energy sources. Wind and solar energy provide public health and environmental benefits to the social. Wind turbines may also reduce the amount of electricity generation from fossil fuels, which results in lower total air pollution and carbon dioxide emissions. In order to better optimize the effect of social energy economic management and facilitate the multiobjective decision making of coordinated development of energy and socioeconomic environment, a modeling and analysis method of economic benefits of wind power generation based on deep learning is proposed. In this paper, based on the principle of deep learning, the evaluation indicators of wind power economic benefits are excavated, a scientific and reasonable economic benefit evaluation system is constructed, a wind power economic benefit analysis model supported by public management is constructed, and the steps of wind power economic benefit analysis are simplified. It is concluded that the modeling and analysis method of wind power economic benefits based on deep learning has high practicability in the actual application process, which is convenient for the prediction and analysis of energy demand for social and economic development.

## 1. Introduction

The economic benefit modeling and analysis method of wind power generation is bound to become the main form of energy development in the future. However, at present, the concept, physical framework, and related models of economic benefit modeling and analysis methods of wind power generation have been deeply studied at home and abroad, but most of the existing studies are based on a specific/assumed regional energy economic data, which is not universal, especially in the current economic benefit modeling and analysis methods of wind power generation. All kinds of physical equipment and their mathematical models have not been combed and summarized, and the theoretical system suitable for the economic benefit evaluation of comprehensive wind power generation has not been established. The analysis of the economic, environmental, and social benefits that energy development and management can bring is still in the conceptual stage. Therefore, based on the relevant research and exploration at home and abroad, this paper optimizes the economic benefit modeling and analysis method of wind power generation based on the deep learning method. Deep learning is the internal law and representation level of learning sample data [1–3]. The information obtained in the learning process is very helpful to the solution of data such as words, images, and sounds. Deep learning is a complex machine learning algorithm. Its effect in speech and image is far better than that of previous related technologies. Deep learning has achieved a lot in data mining, machine learning, translation, natural language, multimedia learning, speech, recommendation, and personal related fields. Deep learning enables machines to imitate human activities such as audio-visual and thinking, identify difficult problems, and make great progress in artificial intelligence-related technologies. In terms of its basic framework, model, and comprehensive benefit evaluation system, this paper summarizes and analyzes the research status and theoretical results at home and abroad, combs the shortcomings of the current research, and looks forward to the key research directions and key problems of wind power generation economic benefit modeling and analysis method modeling and comprehensive benefit evaluation in the future.

## 2. Modeling and Analysis Method of Economic Benefits of Wind Power Generation

Wind power projects aim at the efficient use of wind energy as a new energy. As a clean and renewable energy, wind energy is of great significance to energy conservation and pollution reduction in our society. One of the important features of wind power projects is their significant social benefits. From this perspective, wind energy is a clean and renewable energy source, and also a new type of energy resource that needs to be further developed in the country. The development and utilization of wind energy resources are an effective way to optimize the country's energy structure and implement sustainable energy development, and are also conducive to ecological conservation and environmental protection. After the completion of the wind farm, the wind turbine can provide renewable power generation for the power grid every year, which can help reduce the country's consumption of other energy sources such as standard coal and, in turn, reduce the emissions of a variety of harmful gases and exhausts such as sulfur dioxide, carbon dioxide emissions, soot emissions, carbon monoxide and hydrocarbons, nitrogen oxide, and suspended particulate matter. At the same time, wind power projects can also bring huge social benefits and boost employment. According to statistics, every 1 mW of installed capacity will directly increase employment by 5 people and 20 indirectly. Therefore, besides economic evaluation and social benefit evaluation, it is also necessary to conduct a comprehensive evaluation of wind power construction projects. The content of the index system for social benefit evaluation of wind power construction projects is divided into 3 parts: natural environment impact, social economic impact, and social environmental impact. Using the deep learning-based modeling and analysis method for wind power economic benefits, this paper demonstrates that the cost and benefit of wind power generation are positively correlated with the reliability level, so it can maximize the overall economic and environmental benefits of the wind power generation model, and contribute to social and economic development. It provides an important reference for forecasting and analysis of energy demand.

Wind power construction projects belong to infrastructure construction and are also profitable projects. Compared with other construction projects, wind power construction projects have their own characteristics:

1. From the perspective of construction methods and project operation methods, wind power construction projects are projects that are completed have also been developed and utilized at the same time as primary energy development and construction. Compared with hydropower, thermal power, and nuclear power projects, wind power projects do not involve troubles like the coal mining and transportation required by thermal power, or the investment required by oil. Compared with hydropower, thermal power, and nuclear power projects, the construction period is short, the investment is flexible, the automatic control level is high, and the operation and management personnel are less. After the project is completed, the operation cycle is relatively long.
2. The cost and benefit of wind power construction projects are both very important in the form of financial microscopic cost-effectiveness and national economic macroscopical cost-effectiveness. Wind power construction projects are first and foremost profitable projects, considering their microeconomic benefits. Moreover, wind power projects themselves have significant social benefits. One of the prominent reasons for carrying out wind power construction projects is that this clean energy is renewable and pollution-free energy, and the wind power industry can promote the development of such industries as machinery manufacturing. Therefore, in the process of project construction and evaluation, it is necessary to fully consider the cost-effectiveness of both micro and macro aspects.
3. Wind power construction projects have strict requirements on the construction period. Completion on time is critical to the success or failure of wind power projects. For owners and developers, the importance of timely completion even outweighs the basic goal of making a profit as soon as possible. In many wind power projects, owners and developers are bound by commercial operation deadlines, subject to power purchase agreements or financing agreements. In addition, if the production tax credit policy is applicable to the location of the project, the new project must be put into use before the production tax credit expires. Improperly scheduled engineering schedules can increase recurring expenses. Many factors will cause the project to be delayed in completion, in order to avoid that the project must have a strong ability to resist risks, and have a strict plan for the use of funds and the survival of the project.
4. From the perspective of the benefits and costs of wind power construction projects, due to the limitation of independent manufacturing of wind power equipment in the country, the profitability of such projects is low and the investment recovery period is long. At present, after the completion of the project, the cost of power generation is high and the profit is low, and there is still a profitability gap compared with thermal power projects. At present, the cost of wind power generation in domestic enterprises is significantly higher than that of water and thermal power generation. The investment benefits of wind power construction projects are socially significant. Wind power construction projects not only have economic benefits but also have great social benefits, which can help drive related industries, reduce environmental pollution, and save energy.

Although the construction period of wind power projects is long, the investment is huge, and the construction and installation technologies are high-end and complicated, we should still give priority to utilizing wind energy resources because it can help develop clean energy and optimize the energy structure of a region, support the sustainable development of the regional energy industry, and reduce the pressure on environmental protection. At present, China has completed many large-scale power generation projects, such as the Inner Mongolia 400 mW wind power project of Datang Group, the 135 mW wind power project of Inner Mongolia Chuangyuan Wind Power Co., Ltd., and the 102.5 mW onshore wind farm project in Jiangsu Province. And more will be built. For example, Zhejiang Province will focus on the construction of nine wind power projects in 2022 including seven offshore wind power projects totaling at 2.254 GW. Energy saving and emission reduction, reducing energy consumption, and improving comprehensive utilization of resources are a long-term strategic policy for the country's economic and social development. For a long period of time, the country will attach great importance to sustainable development and promotion of energy conservation, as well as emission reduction while pursuing economic development. At present, although the country has achieved certain achievements in wind power generation, some problems still remain such as the lack of in-depth analysis of environmental impact and low efficiency in wind energy utilization. Therefore, it is necessary to further strengthen the development and utilization of wind power, improve the domestic wind power industry system, and continuously improve key technical capabilities so as to further enhance the economic and environmental benefits of wind power projects.

At this stage, there is relatively little research on the economic benefit modeling and analysis method and benefit evaluation of wind power generation. In the existing research, the benefits of CCHP model and gas turbine model are evaluated, and the model investment cost and primary energy consumption are not selected as the evaluation indexes of economic, energy consumption, and environmental benefits of the economic benefit modeling and analysis method of wind power generation [4]. The economic benefit evaluation index system of wind power generation constructed in this paper covers the economic, social, and environmental benefits that can be brought by the economic benefit modeling and analysis method of wind power generation, but there are few secondary indicators, which cannot fully and deeply reflect the benefits that can be brought by the economic benefit modeling and analysis method of wind power generation. From the energy link, device link, distribution network link, and user link, the benefit evaluation index system of regional wind power generation economic benefit modeling analysis method is established, and the indexes reflecting economic benefit, social benefit, and environmental benefit are integrated into each link. Considering the coupling relationship between the internal economy of the regional wind power generation economic benefit modeling and analysis method can comprehensively reflect the economic, environmental, and social benefits brought by the wind power generation economic benefit modeling and analysis method, but the granularity of the indicators selected by the index system is not fine enough and the benefit indicators covered are not comprehensive enough, as such the load rate of wind power grid is not considered. It also does not take into account economic indicators such as investment income, which still needs to be further enriched and improved. Based on this, the technical and economic indicators (investment and operation cost, net present value NPV, internal rate of return IRR, investment payback period PP, etc.), gas emission reduction indicators, fossil energy consumption, and other indicators of the economic benefit modeling and analysis method of wind power generation are used to measure the investment value and environmental protection benefits of the economic benefit modeling and analysis method of wind power generation, which is concise, clear, and operable.

There are many factors affecting the economy of distributed generation model, which can be divided into two levels: planning level and operation level. The following will analyze the influencing factors from these two levels [5–7]. The objective functions of the existing research on the economic benefit management model of wind energy power generation mainly include the following three categories:

(1) $$\begin{array}{c} \min F\left(C\right)=\overset{N}{\underset{n=1}{\sum }}1-\min C_{n},\\ F\left(B\right)=\overset{M}{\underset{m=1}{\sum }}B_{m}-P,\\ F\left(L\right)=\min\text{F}\left(C\right)\sum F\left(L_{E}\right)+F\left(L_{H}\right)+F\left(L_{G}\right), \end{array}$$

where *F*(*C*) represents the model cost function; *C*_*n*_ represents each cost item; minf *C*_*n*_ represents the model fuel consumption function; *P* represents the fuel consumption parameters of each unit; *F*(*L*_*E*_) represents the energy shortage function of the model; and *F*(*L*_*H*_) and *F*(*L*_*G*_) represent the power off, heat off, and gas off functions of the model, respectively. At the same time, when the economic benefit analysis model of wind power generation is used for data scheduling control, the constraints that need to be considered include the physical and economic data constraints of various submodels such as power, heat, and natural gas, which is more complex than the traditional independent scheduling method of power, natural gas, and heat. The mathematical expression is as follows:

(2) $$\begin{array}{c} \min\text{F}=\frac{F\left(B\right)-F\left(L\right)}{R\left(F_{1}\left(P\left(t\right)\right),F_{2}\left(P\left(v\right)\right)\right)}, \end{array}$$

where *P*(*t*) is the number of switchboard groups, and *t* is the scheduling cycle. *P*(*v*) Is the planned output vector of each unit in period *R*, and the environmental economic regulation model often contains multiple objectives, which are often contradictory and conflicting with each other. Improving the performance of one target may reduce the performance of other targets. In other words, there is no solution that can ensure the optimal economic cost and environmental protection at the same time, so they can only be compromised and coordinated. The process of solving the multiobjective optimization problem is to find a set of decision vectors that meet the noninferiority and constraints of all objective functions and the set of corresponding objective function values, that is, the optimal solution of economic benefits, so that the decision maker can determine the acceptable decision-making state and corresponding objective function values according to the utility function or preference [7–9]. The economic decision making of wind power generation based on deep learning is the basis and basis to guide safety activities. Selecting a reasonable scheme from several feasible safety investment schemes requires technical and economic analysis and evaluation. This paper adopts the “benefit-cost” analysis and decision-making method. The steps of safety investment scheme decision making are as follows: we calculate the effect of investment scheme

(3) $$\begin{array}{c} \Delta R=\min F\prod U\times P, \end{array}$$

where Δ*R* is effect of investment scheme [8, 10–13]; *U* is accident loss and is expected probability. We calculate the benefits of safety investment scheme

(4) $$\begin{array}{c} \Delta B=\cap \Delta R\left(R_{0}-R_{1}\right), \end{array}$$

where Δ*B* is benefits of the investment scheme; *R*_0_ is effect before the implementation of the investment scheme; and *R*_1_ is effect after the implementation of the investment scheme. We calculate the benefit of safety investment

(5) $$\begin{array}{c} E=\Delta B-\frac{1}{C}. \end{array}$$

In-depth education theory, the state space method is used to describe the model in time domain. The equation of state of the model can be described as

(6) $$\begin{array}{c} x=\text{Ef}\left(u,t\right)-R^{m}R^{r}, \end{array}$$

where *R*^*m*^*R*^*r*^ are the Euclidean space, vector *r* is the m-dimension, and *u* is the *t* dimension. For simplicity, we take the first-order steady-state free model as an example. At this time, *M* = 1r0, set *l* as the state of the model, and F as the control strategy function [14]. Polynomial fitting is used to obtain

(7) $$\begin{array}{c} \frac{\text{d}L}{\text{d}t}=f\left(L\right)=a_{0}+a_{1}L+a_{2}L^{2}. \end{array}$$

The economic model of wind power generation based on deep learning is a complex model composed of safety investment resources, safety investment structure, safety model and its generated model, safety state, and safety benefits.

Feedback and delay in the economic model of wind power generation are based on deep learning. The concept of deep learning was first introduced by Hinton et al. in 2006, which refers to the machine learning process of obtaining a deep network structure containing multiple levels through a certain training method based on sample data. The traditional neural network randomly initializes the weights in the network, which makes the network easy to converge to the local minimum value. To solve this problem, Hinton proposes to use the unsupervised pretraining method to optimize the initial value of the network weights and then fine-tune the weights. The importance of deep learning in academia and industry is becoming more and more prominent, and deep learning has achieved obvious advantages in different application fields. Deep learning is a new research direction in the field of machine learning. In recent years, breakthroughs have been made in various applications such as speech recognition and computer vision. The motivation is to establish a model to simulate the neural connection structure of the human brain. When processing signals such as images, sounds, and texts, the data features are described hierarchically through multiple transformation stages, and then, the data interpretation is given. Deep learning combines low-level features to form more abstract high-level representations, attribute categories or features, and give hierarchical feature representations of data. In models learned by deep learning, there are more levels of nonlinear operations. Deep learning transforms the feature representation of the sample in the original space into a new feature space by performing layer-by-layer feature transformation on the original signal, and automatically learns to obtain a hierarchical feature representation, which is more conducive to classification or feature visualization. Based on the application of deep learning technology, by learning the implicit representation of users and items from massive data, and then building a recommendation model, an effective recommendation list is finally generated to users. Compared with traditional recommender systems, deep learning-based recommender systems can use deep learning technology to automatically learn abstract hidden features of users and items by fusing various types of multisource heterogeneous data and model sequential patterns in user behavior. It can more effectively reflect the different preferences of users and improve the accuracy of recommendation. The current deep learning recommendation system needs to model many elements, including not only the interaction data between users and items but also the spatiotemporal sequence patterns of user behavior, the influence of social relations, the dynamic evolution of user preferences, and the dynamics of item characteristics. And changes to more modeling elements can improve the performance of the recommender system. Therefore, researching new deep learning architectures that can express and integrate multiple elements is also one of the future research directions. In addition to directly displaying the recommendation results, deep learning-based recommendation systems often also display appropriate recommendation reasons to tell users why the system thinks such a recommendation is reasonable. Improving the interpretability of the recommendation system can improve the user's acceptance of the recommendation results and also improve the user's experience in system transparency, credibility, distinguishability, effectiveness, and satisfaction. The end-to-end model directly uses multisource heterogeneous data as input to predict the user's preference for items. The result of model training is to give the structure of the deep neural network and the connection weights between neurons, so as to optimize the data, model, and economic significance, as well as to research at the level to improve the interpretability based on deep learning technology.

According to the principle of deep education theory, the feedback loop is the basic structure of the model. The feedback phenomenon in the economic model of wind power generation based on deep learning is very common. The change of safety investment structure and strength will inevitably lead to the change of the overall safety state of the safety model. This change will affect the supply through the feedback of increasing or reducing the supply of safety resources in response to the control mechanism of accident risk [15–17]. This constitutes the feedback loop in the economic model of wind power generation, as shown in Figure 1.

The safety investment based on deep learning is oriented to the model elements of human, material, environment, and management in the model. The influence of these elements themselves and their interaction on the safety state of the model is very complex. Therefore, the safety investment must go deep into the model structure and adjust the investment proportion and structure of safety resources from different angles [18]. We ensure the full utilization of enterprise safety resources and maximize safety benefits. The essence of the in-depth education theory of the economic decision-making of wind power generation is to obtain the model function results by simulating the structure of the economic model of wind power generation. When the deviation between the results and the target value is too large, the decision maker will consider changing the safe resource investment allocation scheme to reduce the deviation until the satisfactory simulation results are obtained, or by simulating the resource allocation structure of different wind power generation economic models, the optimal decision-making scheme can be selected.

Under the condition of meeting the economic operation constraints of wind power generation and taking into account the objectives of economic benefits and environmental protection, the economic benefit model of wind power generation is mainly used to realize the reasonable load distribution among the power generation units in the power model. However, in the power model composed of several traditional thermal power units and wind farms, the inherent intermittence and uncertainty of wind energy will interfere with the actual dispatching. In order to reduce adverse effects, it is necessary to consider the standby penalty factors caused by the planned output of the wind farm exceeding or lower than the actual output in terms of economic benefits and environmental protection, and eliminate the interference data based on deep learning technology. Specifically, if the planned output of the wind farm exceeds the actual output, the difference between the planned value and the actual value needs to be purchased from other power models; otherwise, the power balance cannot be achieved within this model. That is, overestimating the output of wind power will bring additional power generation costs and benefits of wind power generation, so it is necessary to introduce corresponding standby mechanism. On the contrary, if the planned output of the wind farm is lower than the actual output, it will cause the waste of power exceeding the planned value in the actual value. At the same time, in order to achieve power balance, traditional thermal power units undertake the power generation task that they do not need to undertake, so as to reduce unnecessary power generation costs and improve the efficiency of wind power generation. Therefore, it is necessary to introduce the corresponding punishment mechanism. Based on the above discussion, the economic scheduling of the wind power grid-connected power model is regarded as a multiobjective stochastic programming problem. Considering the uncertainty of wind power and other necessary constraints, we strive to minimize the overall generation cost and wind power generation benefit of the model, and then explore the optimal load distribution between conventional thermal power units and wind farms. The minimization of power generation cost in power model can be expressed as follows:

(8) $$\begin{array}{c} \min F_{1}=\min\left\{\overset{M}{\underset{i=1}{\sum }}C_{i}\left(T_{i}\right)+\overset{N}{\underset{i=1}{\sum }}C_{w,i}\left(W_{i}\right)+\overset{N}{\underset{i=1}{\sum }}C_{p,i}\left(W_{r,i}-W_{i}\right)-\frac{\text{d}L}{\text{d}t}\right\}, \end{array}$$

where *W*_*i*_ is the number of thermal motor units, *W*_*r*,*i*_ is the number of wind turbine units in the wind farm, *C*_*p*,*i*_ is planned output of the *i*th thermal power unit, *C*_*i*_ is the planned output of the *i*th wind turbine, and *C*_*w*,*i*_ is the actual output of the *i*th wind turbine, which is a random variable subject to a specific probability distribution. Its variation range is 0 ≤ W1 ≤ WA, and wad is the rated power of the *i*th wind turbine. CO is the cost function of the *i*th thermal power unit. CO is the explicit cost function of the *i*th wind turbine, and its value is related to the ownership of the wind farm. CNO is the penalty cost function caused by underestimating the actual output of the *i*th wind turbine; on the contrary, CO is the standby cost function caused by overestimating the actual output of the *i*th wind turbine. The power generation cost of thermal power unit considering valve point effect is

(9) $$\begin{array}{c} C_{i}\left(T_{i}\right)=\frac{a_{i}}{2\min F_{1}}+b_{i}d_{i}+\left|e_{i}\sin\left(f_{i}\left(T_{i,\min}-T_{i}\right)\right)\right|, \end{array}$$

where *a*_*i*_, *b*_*i*_, *d*_*i*_, and *e*_*i*_ are power generation cost coefficients; *f*_*i*_(*T*_*i*,min_ − *T*_*i*_) is the lower limit of active power output of the *i*th thermal power unit. In order to reduce the computational complexity of the algorithm and improve the computational speed, a nondominated set ranking method is proposed to realize population classification. In order to reflect more intuitively, the table lists the single objective optimization extremum of minimum economic cost and wind power generation benefit at the frontier endpoint under different confidence levels in Table 1.

According to the analysis and calculation results in the table, with the increase of the confidence level in meeting the constraints, the total output of conventional units in the power model decreases monotonously, and the output of wind farm increases accordingly. This shows that although the increase of the proportion of wind farm output in the power model is conducive to economy and environmental protection, it also brings greater risks to the operation of the model. If only economic benefits are considered, when the dispatching scheme with the lowest economic cost is selected, the benefit of wind power generation will increase, which is not conducive to environmental protection. If only environmental protection is considered, when the dispatching scheme with the least benefit of wind power generation is selected, the power generation cost will be increased, which is not conducive to economy. Therefore, it is necessary to integrate various factors and fully mine the information contained in the optimal set, so as to provide reasonable decision-making scheme for power model dispatchers and realize the construction goal of wind power generation household benefit model.

The safeguard measures for the implementation of wind power projects are divided into three stages: safeguard measures before construction, during construction, and after construction. The measures before construction include organizational safeguards, material and equipment safeguards, contract safeguards, and system safeguards. The ones during the construction include technical safeguards and safety safeguards. And the ones after construction mainly include data and information guarantee and the incentive mechanism. The deep learning-based wind power economic benefit modeling and analysis method established in this paper also include a feedback mechanism, which affects the supply by increasing or decreasing the feedback of the supply of safety resources to control the accident risk. The economic dispatch of wind power grid-connected model is regarded as a multiobjective stochastic programming problem, considering the uncertainty of wind power and other necessary constraints, and strive to minimize the overall power generation cost and wind power generation benefit of the model, and then explore conventional thermal power units and wind farms, as well as optimal load distribution among them. Through simulation, operation optimization, and benefit evaluation, it plays a real guiding role in evaluating the risk and benefit of wind power project investment. At the same time, combined with the actual application, the program is continuously improved and perfected to make it more applicable and scientific.

## 3. Analysis of Experimental Results

In order to verify the practical application effect of the economic benefit modeling and analysis method of wind power generation based on deep learning, the experimental detection is carried out. Firstly, the new configuration of wind power generation is optimized, and a benchmark value is set for the experimental parameters. The details are shown in Table 2.

From the above table, the economic benefits of wind resources and light resources show certain complementary characteristics, but the impact of this complementary characteristic on the economic benefit analysis model needs further analysis. Whether the economic benefits of scenery resources are complementary is mainly reflected in whether the reliability of the model can be improved. The reliability of the wind and solar energy economic benefit complementary model is compared with that of the wind turbine model and the photovoltaic economic benefit model. The comparison results are shown in Table 3.

According to the first mock examination, the economic benefits of wind power generation based on deep learning are less than that of traditional single models, which is much better than the single power generation model. The comparison results fully show that wind solar complementary power generation has complementary advantages. In order to explore the reliability of the model, the relationship between the total generation cost and economic benefits of the power model in each period is compared. It can be found from the table that in each period, the power generation cost after considering both reliability constraints and effectiveness constraints is lower than that considering reliability alone in Table 4.

In order to explore the impact of different optimization objectives on power model dispatching decision making based on economic cost and wind power generation benefit under uncertainty, the wind power generation economic benefit models constructed in this paper are transformed into the following forms: the objective function is divided into single objective and multiobjective, while the constraints remain unchanged. Accordingly, the optimal planned output per unit period obtained by the dynamic economic dispatching model under uncertainty is shown in Table 5.

The generation cost obtained by the constraint is higher than that obtained by considering the effectiveness constraint alone. In addition, in terms of emission protection, the table also compares the relationship between the reliability and effectiveness of the power economic consumption model. Combined with the table, we can draw the following conclusions: strengthening the reliability constraint will increase the power generation cost and wind power generation benefit of the power model, while strengthening the effectiveness constraint will reduce the power generation cost and improve the wind power generation benefit as shown in Figures 2 and 3.

In the financial evaluation of construction projects, in order to describe and characterize the complex economic effects of the project from different angles and aspects, a variety of evaluation indicators have been designed. These indicators have their own advantages and disadvantages. In project evaluation, it is difficult to fully reflect the full picture of the project's economic effects by using only one or two indicators. Therefore, we should have an optimization index system that can basically describe the economic effects of the project more objectively and scientifically from all aspects so that we can correctly judge the feasibility of the project and correctly select the optimization index system. In the economic evaluation, according to the characteristics of wind power construction projects, the economic benefit model based on deep learning is mainly to meet the economic operation constraints of wind power generation, taking into account the goals of economic benefits and environmental protection. The economic decision making of wind power generation based on deep learning is the basis for guiding safety activities. To choose a reasonable one from several feasible safe investment schemes, it is necessary to carry out technical and economic analysis and evaluation. This paper adopts the “benefit-cost” analysis and decision-making method. The model function results are obtained by simulating the structure of the wind power economic model. When the deviation between the result and the target value is too large, the decision maker will consider changing the safe resource investment allocation plan to reduce the deviation until a satisfactory simulation result is obtained, or by simulating the resource allocation structure of different wind power economic models, and then select the optimal decision plan.

To sum up, the power generation cost and benefit of wind power generation are positively correlated with the reliability level. Based on the positive correlation characteristics of this period, it is confirmed that the proposed economic benefit model of wind power generation based on deep school can effectively control the economic loss of wind power generation, reduce the emission loss of wind power generation, realize the integrated management of the economic benefits of wind power generation, and maximize the overall economic and environmental benefits of the wind power generation model.

## 4. Conclusion

With the continuous development and application of new technologies and new equipment, the basic framework of economic benefit modeling and analysis method of wind power generation is also progressing and evolving, and its economic, environmental, and social benefits will be increasingly obvious. Under the background of the deepening theoretical research on the economic benefit modeling and analysis method of wind power generation in China and the orderly implementation of pilot projects, the modeling and simulation, operation optimization, and benefit evaluation of the economic benefit modeling and analysis method of wind power generation have good implementation conditions, which is the key direction for further research in the future. Based on the research on the basic framework of the economic benefit modeling and analysis method of wind power generation, the physical and economic modeling, and benefit evaluation system of independent and coupled equipment units, this paper aims to clarify the physical boundary and benefit of the planning, construction, and operation control of the economic benefit modeling and analysis method of wind power generation, so as to provide reference for the landing of relevant projects and the research and development of simulation platform. With the rapid economic development, the country's demand for energy is increasing. Wind resources, as a renewable energy, clean and pollution-free, have huge environmental benefits and can be used to improve the energy structure, promote technological progress, and realize a low-carbon economy. Wind resources are widely distributed and the cost of power generation is low, thus having rich economic benefits. In order to meet the electricity demand for its economic and social development, the state encourages the development of wind power, and China's wind power construction has broad prospects. The country has rich wind resources, and the potential for development is 1 billion kilowatts. China's wind resources are mainly concentrated in the grasslands in the north, northwest, and northeast regions, as well as the coastal areas and islands in the east and southeast. It is of great significance to analyze the economic benefits and environmental impact of wind power construction projects to accelerate the development of wind power generation. Firstly, it can help ensure the smooth implementation of the country's sustainable development strategy. With the continuous development of science and technology, it has become more and more important for the country to keep a balance between economic development and environmental protection. The implementation of sustainable development has become a basic policy for the country's national economic and social development. When pursuing sustainable development, environmental protection and economic development must be coordinated. Many wind farms have been built in China, and although wind power projects do not produce industrial wastes and other pollutants, they will cause a series of negative impacts such as noise pollution, vegetation damage, and impact on ecosystems to varying degrees. Therefore, from the beginning of construction, full consideration must be given to the prevention and control of the abovementioned impacts to guarantee the implementation of sustainable development strategy, and realize environmental benefits while creating economic benefits. Secondly, economic benefit is the top concern for wind farm construction, and the evaluation based on deep learning is essential for decision making of wind power construction projects.

## Figures and Tables

**Figure 1:** Causal feedback diagram of energy economy security investment function based on deep learning.

**Figure 2:** Broken line of power generation cost-benefit under different constraints.

**Figure 3:** Broken line diagram of wind power generation benefits under different constraints.

**Table 1:** Cost benefit extremum under different confidence levels.

	(*η*1 = *η*2 = *η*3 = 0.1)			(*η*1 = *η*2 = *η*3 = 0.15)		
	Economic optimum	Optimal protection	Environmental	Economic optimum	Optimal protection	Environmental
Economic cost (s)	2560500	2576900		2326700	2342000	
Pollutant emission (IB)	305350	303290		247590	244870	

**Table 2:** Basic values of experimental parameters.

Symbol	Company	Numerical value
Pw	Yuan (kW)	4900
Ps	Yuan (kW)	6100
Nw	Yuan (kW)	120
Ns	Yuan (kW)	20
Qcxin	Yuan (kW)	0.63
Qxing	Yuan (kWh)	1.0
Zw	Yuan (kWh)	0.2
Zs	Yuan (kWh)	0.43
Lw	year	30
v	—	0.15
Yzng	Yuan (kW)	500
Yxiag	Yuan (kW)	460
Tz	Yuan (kW)	20000
Qcgin	Yuan (kWh)	0.49
Qxiag	Yuan (kWh)	13
Qzign	Yuan (kWh)	0.08

**Table 3:** Comparison of reliability indexes.

System type	Pw (kW)	Ps (kW)	Economic performance (%)
Paper model	2.215 × 10^4^	3.798 × 10^4^	15.65
Fan model	3.248 × 10^4^	—	7.18
Wind solar complementary model	—	2.298 × 10^4^	2.88

**Table 4:** Total cost-effectiveness of each period under different constraints.

Time interval	Cost			Discharge		
	Effectiveness	Reliability and effectiveness	Reliability	Effectiveness	Reliability and effectiveness	Reliability
A	7565.65	7526.65	8958.65	482.60	496.65	625.33
B	6215.85	8562.32	10525	325.65	585.65	652.62
C	7932.52	8654.62	9536.35	521.65	598.62	628.9
D	8565.5	8571.6	12365.65	476.65	756.32	865.35
E	7725.32	10365.65	11526.65	532.65	772.65	929.65
F	11263.65	10325.65	18652.32	956.65	1214.65	2282.65
G	10856.65	12958.25	16256.32	1141.65	1225.32	1765.65
H	11236.25	14523.25	15325.65	6523.65	1252.32	1298.85
I	12.6458	14352.65	15325.65	1562.52	1165.02	1885.65
J	11352.65	14652.65	15653.85	758.65	1252.65	1086.65
K	14365.25	15652.65	19353.65	1568.65	1552.65	3256.65

**Table 5:** Optimal constraint plan (mW) in each period obtained by dynamic economic dispatching model.

Time	Machine 1	Machine 2	Machine 3	Machine 4	Machine 5	Machine 6
*A*	189.65	46.85	81.6	122.32	62.32	58.65
*B*	99.25	201.86	75.32	132.5	68.65	46.8
*C*	135.65	142.65	75.65	165.63	72.35	47.62
*D*	178.65	86.65	110.65	204.65	126.52	63.65
*E*	101.65	200.32	98.5	202.98	90.55	48.65

## Data Availability

The datasets used or analyzed during the current study are available from the corresponding author upon reasonable request.
